This article has been retracted.

# *Potamogeton perfoliatus* L. Extract Attenuates Neuroinflammation and Neuropathic Pain in Sciatic Nerve Chronic Constriction Injury-Induced Peripheral Neuropathy in Rats

**DOI:** 10.3389/fphar.2021.799444

**Published:** 2021-12-20

**Authors:** Mona F. Mahmoud, Samar Rezq, Amira E. Alsemeh, Mohamed A. O. Abdelfattah, Assem M. El-Shazly, Rachid Daoud, Mohamed A. El Raey, Mansour Sobeh

**Affiliations:** ^1^ Department of Pharmacology and Toxicology, Faculty of Pharmacy, Zagazig University, Zagazig, Egypt; ^2^ Department of Anatomy and Embryology, Faculty of Medicine, Zagazig University, Zagazig, Egypt; ^3^ College of Engineering and Technology, American University of the Middle East, Egaila, Kuwait; ^4^ Department of Pharmacognosy, Faculty of Pharmacy, Zagazig University, Zagazig, Egypt; ^5^ African Genome Center, Mohammed VI Polytechnic University (UM6P), Ben Guerir, Morocco; ^6^ Department of Phytochemistry and Plant Systematics, Pharmaceutical Division, National Research Centre, Dokki, Cairo, Egypt; ^7^ AgroBioSciences Research, Mohammed VI Polytechnic University, Ben-Guerir, Morocco

**Keywords:** Potamogeton perfoliatus, chronic constriction injury, CD68, GFAP, iNOS

## Abstract

Sciatic nerve injury is often associated with neuropathic pain and neuroinflammation in the central and peripheral nervous systems. In our previous work, *Potamogeton perfoliatus* L. displayed anti-inflammatory, antipyretic and analgesic properties, predominantly via the inhibition of COX-2 enzyme and attenuation of oxidative stress. Herein, we extended our investigations to study the effects of the plant’s extract on pain-related behaviors, oxidative stress, apoptosis markers, GFAP, CD68 and neuro-inflammation in sciatic nerve chronic constriction injury (CCI) rat model. The levels of the pro-inflammatory marker proteins in sciatic nerve and brainstem were measured with ELISA 14 days after CCI induction. Pretreatment with the extract significantly attenuated mechanical and cold allodynia and heat hyperalgesia with better potential than the reference drug, pregabalin. In addition, CCI lead to the overexpression of prostaglandin E2 (PGE2), inducible nitric oxide synthase (iNOS), tumor necrosis alpha (TNFα), nuclear factor κB (NF-κB), cyclooxygenase-2 (COX-2), 5-lipoxygenase (5-LOX), and NADPH oxidase-1 (NOX-1) and decreased the catalase level in sciatic nerve and brainstem. The observed neuro-inflammatory changes were accompanied with glial cells activation (increased GFAP and CD68 positive cells), apoptosis (increased Bax) and structural changes in both brainstem and sciatic nerve. The studied extract attenuated the CCI-induced neuro-inflammatory changes, oxidative stress, and apoptosis while it induced the expression of Bcl-2 and catalase in a dose dependent manner. It also decreased the brainstem expression of CD68 and GFAP indicating a possible neuroprotection effect. Taking together, *P. perfoliatus* may be considered as a novel therapy for neuropathic pain patients after performing the required clinical trials.

## Introduction

Neuropathic pain is widely described as burning or electrical like sensation that affects mainly the areas sensitive to touch. The pain is associated with many pathological conditions including neuralgia, stroke, diabetic neuropathy, cancer, herpes zoster infection, and multiple sclerosis, among others. Neuropathic pain is mainly caused by an ailment or a lesion in the somatosensory nervous system, which mediates the perception of temperature, pressure, pain, position, and touch (Costigan et al., 2009; Sobeh et al., 2019).

Hyperalgesia and allodynia are two classic symptoms of neuropathic pain. The former is defined as an increased sensitivity towards a painful stimulus, while the later denotes a painful sensation to a stimulus that is normally non-painful (Zimmermann 2001; Sobeh et al., 2020). The symptoms of neuropathic pain are always manifested as excruciating pain aggravated upon pressure, pins and needles sensation, numbness, and difficulty in sensing temperatures properly (Woolf and Mannion, 1999).

Management of the condition depends mainly on relieving the symptoms rather than eliminating the causative, which is rarely possible. Patients do not usually respond to the commonly used analgesics and non-steroidal anti-inflammatory drugs (NSAIDs) as neuropathic pain is entirely different from the inflammatory pain associated with some chronic conditions such as rheumatoid arthritis for example (Dworkin et al., 2007).

Antidepressants such as the tricyclic amitriptyline or the serotonin-norepinephrine reuptake inhibitor duloxetine were proven effective in numerous neuropathic pain conditions. Some antiepileptic drugs such as gabapentin and pregabalin are also involved in the management of neuropathic pain by virtue of their potential to bind to the voltage gated Ca^2+^ channels leading to a decrease in sensitization followed by an analgesic effect. However, majority of these treatments have moderate efficacy and diverse side effects, which imposes high demand for novel alternatives (Sindrup and Jensen, 1999). Secondary metabolites isolated from various medicinal plants have been used in traditional medicine to relieve the pain associated with many pathological conditions and could represent safer alternatives for managing neuropathic pain (Van Wyk and Wink, 2015; Rezq et al., 2020).

Potamogetonaceae, or the pondweed family, includes 110 species belonging to six genera, where the genus *Potamogeton* is the largest among them. The usage of various plants from this genus in folk medicine is reported for curing several pathological conditions (Shirshova et al., 2012). The perennial hydrophyte, *Potamogeton perfoliatus* L., known as the redhead grass, is found in many flowing and standing freshwater habitats in almost all the continents but not in South America. Several secondary metabolites from different chemical classes were identified in *P. perfoliatus*, among them flavonoids and fatty acids. Recently, we have characterized the phytochemical profile of *P. perfoliatus* using HPLC-MS and it furnished 15 secondary metabolites. These include several phenolic acids (*p*-coumaric acid, *p*-hydroxybenzoic acid, and syringic acid), iridoid (catalpol sulphate), and flavonoids (luteolin glucoside, quercetin glucoside and rosmarinic acid). We also examined its analgesic, anti-inflammatory, and antipyretic activities (Rezq et al., 2021).

Prolonged peripheral nerve injury leads to increase in peripheral nerves and spinal cord synaptic networks ectopic activity. Moreover, the descending brainstem nociceptive circuits to the spinal cord are activated and hence play an essential role in the severity of the neuropathic pain-related behavior (Suzuki et al., 2002). Therefore, targeting the mechanisms involved in peripheral, spinal and supraspinal pathologies observed in neuropathic pain is equally important (Suzuki and Dickenson, 2005). In the current work, we investigated the potential of a bioactive extract from *P. perfoliatus* to attenuate the neuropathic pain induced following a chronic constriction injury (CCI) in the sciatic nerve in rats via evaluating the hyperalgesia and allodynia symptoms. In addition, several pro-inflammatory, oxidative stress, and apoptosis protein markers were measured on the peripheral (sciatic nerve) and supraspinal (brainstem) levels to get some insights about the possible mechanisms through which the extract exerts its effect. Molecular docking at Bcl-2: BH3 interface was used as well to evaluate the anti-apoptotic potential of the extract’s major components. Moreover, histopathological study was conducted to investigate the major structural changes in sciatic nerve and brainstem following CCI and evaluate the extract’s potential to attenuate such changes.

## Materials and Methods

### Plant Material and Extraction

The whole plant, *P. perfoliatus* L., was collected from the Nile River, Zifta, Gharbia governorate, Egypt. Apart from the roots, the plant was cleaned using tap water and air dried. About 500 g was extracted using boiling water (5 L). The filtrate was evaporated using reduced pressure to 300 ml and cleaned several times using ethanol until no precipitate was detected. The soluble aqueous ethanol extract was then evaporated to dryness to yield 38 g (Rezq et al., 2021).

### Animals

Experimental procedure came in accordance with the ethical Guidelines for Animal use and care of the Zagazig University following the National Institute of Health guidelines. Male Wistar rats (n = 36, 8 weeks old; body weight 250–280 g; Faculty of Veterinary Medicine, Zagazig, Egypt) were housed under constant laboratory environment. Animals were maintained on a 12:12 h light-dark cycle and were given ad libitum access to water and chow.

### Chronic Constriction Injury

Induction of CCI in the right sciatic nerve was performed under anesthesia with thiopental sodium (50 mg/kg). An incision was made in the right mid-thigh to expose the common sciatic nerve and the ligation was performed by four loose gut sutures 1 mm apart around the nerve as previously described (Rezq et al., 2020).

### Experimental Design

Animals were randomly divided into six experimental groups (n = 6): control, sham, CCI, CCI treated with the extract (200 and 400 mg/kg) and CCI treated with pregabalin (30 mg/kg) (Wang et al., 2016). Control, sham and CCI groups were given 5 ml/kg (by oral gavage) acacia gum solution (10% w/v), the vehicle used for both the extract and pregabalin. Pregabalin is used in neuropathic pain models in doses that ranges from 3–30 mg/kg (Han et al., 2007; Hahm et al., 2012; Kaur et al., 2015; Sobeh et al., 2019; Yuan et al., 2019; Rezq et al., 2020) with ED50 of 3.3 mg (Hahm et al., 2012). Accordingly, we used a high dose of pregabalin (30 mg/kg) to achieve maximum drug efficacy against our model of neuropathic pain. All treatments were administered for 14 days starting from the first day following the induction of CCI in the sciatic nerve. Behavioral tests were performed on days 1, 7 and 14 following the procedure. Biochemical and histopathological studies were performed at the end of the study (Rezq et al., 2020). The animal number per experiment was calculated using GraphPad StatMate two statistical program. A sample size of six in each group has an 80% power to detect differences of 1.79–3 0.59 (for behavioral tests) and 0.90–2.69 (for the immunohistochemical analysis) and five in each group to detect a difference of 10.07–40.26 (for biochemical assays), between means at alpha of 0.05 (two-tailed).

### Behavioral Tests

As reported in our previous study (Rezq et al., 2020), behavioral tests were performed on day 1, 7 and 14 after the surgery. According to the previously established methods, the following tests were performed:

#### Thermal Hyperalgesia

Thermal hyperalgesia was evaluated using the hot plate test as previously described (Muthuraman and Singh, 2011). Rats were placed on a hot plate, maintained at a temperature of 52.5°C ± 1.0°C. Heat-induced nociceptive behavior was estimated by calculating the latency of paw withdrawal with a cut-off time of 20 s.

#### Mechanical Hyperalgesia (Pinprick Test)

The mid-plantar surface of the injured hind paw was exposed to a gentle force using a bent gauge to avoid skin damage. Paw withdrawal latency was recorded in seconds. The brief normal response was given a value of 0.5 s and the cut-off point was set at 20 s (Hegazy et al., 2020).

#### Acetone Drop Test (Paw Cold-Allodynia)

The cold-allodynia responses were evaluated in animals by exposing the injured paw to acetone spray (100 μl). The response was graded as follows: 0, no response; 1, quick withdrawal or flick of the paw; 2, prolonged withdrawal or repeated flicking; and 3, repeated flicking and paw licking. The final score is the sum of the scores obtained from three different trials (5 min apart) where 0 and nine represent the minimum and maximum scores, respectively (Sobeh et al., 2020).

#### Paint-Brush Test (Mechanical Dynamic Allodynia)

The response of the animals in the different groups to CCI-induced dynamic allodynia was tested using a smooth paintbrush. Briefly, the plantar area of the injured paw was gently rubbed five times with 5 seconds intervals and the number of withdrawals was recorded (0–5). The test was repeated three times (5 min apart). The final score is the sum of the scores obtained from three different trials with a minimum value of 0 and maximum of 15 (Sobeh et al., 2019).

### Tissue Sampling

At day 14 following the CCI induction surgery, the animals were deeply anesthetized and had their sciatic nerve and brainstem removed. For the sciatic nerve, approximately 10 mm piece including the injured site and 5 mm of the surrounding tissues on both sides was dissected. For the brainstem, the medulla oblongata of the brainstem was isolated and cut into two symmetrical parts. We used the medulla oblongata as it contains the rostral ventrolateral medulla (RVM), a major nucleus that is rich in the neurons highly involved in facilitating descending pain transmission inputs to the spinal cord (Vanegas and Schaible, 2004). One part of both tissues was frozen in liquid nitrogen and stored at −80°C while the other part was kept in buffered formalin for the histopathological and immunohistochemical studies.

### Biochemical Analysis

Brainstem and sciatic nerve tissues were homogenized in PBS (10 mg tissue to 100 μl PBS) before being centrifuged for 20 min at 4°C and 14,000 rpm. Bradford test (Bio-Rad, Hercules, CA, United States) was used to determine the protein level in the supernatant used for the biochemical determinations. Rat ELISA Kits from Mybiosource (San Diego, CA, United States) and Cayman (Ann Arbor, Michigan, United States) were used to measure the inducible nitric oxide synthase (iNOS, Cat. #MBS023874) and prostaglandin E2 (PGE2, Cat. # 514,010), respectively. NADPH oxidase 1 (NOX1, Cat. #CSB-EL015959RA), cyclooxygenase-2 (COX-2, Cat. #CSB-E13399r), 5-lipoxygenase (5-LOX, Cat. #CSB-E16982r), catalase (Cat. #CSB-E13439r), TNF-α (Cat. #CSB-E11987r), and NF-κB (Cat. #CSB-E13148r) were all tested using Cusabio (Houston, TX, United States) ELISA Kits according to the manufacturer’s instructions.

### Histopathological Study

Histopathological study was performed on both sciatic nerve and brainstem (medulla oblongata) tissues as previously reported (Bancroft John and Gamble, 2008). Tissues collected from six animals were fixed in 4% paraformaldehyde in 0.1 M phosphate buffer overnight at 4°C and then embedded in paraffin. They were cut into sections of 3 μm thickness and mounted on glass slides, deparaffinized in xylene and stained with hematoxylin and eosin stain (H and E).

### Immunohistochemistry

Tissues of 3 μm thickness were subjected to immunohistochemical staining using the antibodies for Bax (1:100; Santa Cruz Biotechnology, TX, USA), Bcl2 (1:20, clone 124, Dako Corporation, CA, United States), CD68 (1:200; Leica Biosystems Newcastle Ltd., Newcastle, United Kingdom), and glial fibrillary acidic protein (GFAP, 1:100, Abcam, Cambridge, United Kingdom). All stained slides were analysed by light microscopy (LEICA ICC50 W) in the Image Analysis Unit of the Anatomy and Embryology Department, Zagazig University. For morphometrical analyses, the quantitation was done using ImageJ analysis software (Fiji ImageJ; 1.51 n, NIH, United States) (N = 6). The immunohistochemistry (IHC) profiler plugin was used to detect the percentage of positive areas (areas stained with brown colour) to the total area according to the method previously described (Li et al., 2011).

### Data Analysis

Data are presented as mean ± standard error of the mean (SEM). One-way ANOVA or repeated-measures analysis of variance (RM-ANOVA) followed by Tukey post hoc test was used for the statistical comparison between the experimental groups. A significant difference was assumed for values of *p* < 0.05. All statistical tests were performed using Graph pad prism software, version 8 (GraphPad Software Inc., La Jolla, CA, United States).

## Results

### The Extract Attenuates Sciatic Nerve CCI-Induced Heat Hyperalgesia and Cold Allodynia in Rats

In our study, animals with CCI in sciatic nerve showed reduction in the withdrawal latency to heat and increased cold allodynia scores on days 7 and 14 following the surgery (Figures 1A,B) compared to the sham group. Rats treated with 200 and 400 mg/kg of the extract showed restoration of normal heat response latency and cold allodynia responses when evaluated on days 7 and 14 post CCI. Interestingly, the extract at both dose levels (200 and 400 mg/kg) showed better effects on day 14 for heat hyperalgesia and on days 7 and 14 for cold allodynia responses than the standard drug pregabalin (Figure 1).

**FIGURE 1:** *P. perfoliatus* (Pot) extract attenuates the development of heat hyperalgesia and cold allodynia, induced by sciatic nerve chronic constriction injury (CCI). Data are presented as means ± SEM (n = 6/group). Statistical analysis was performed using RM-ANOVA, followed by Tukey post hoc test. The different symbols indicate the significance differences at *p* < 0.05 when compared with sham group (*), CCI group (^#^), and pregabalin group (^@^) at the different time points as indicated in the materials and methods section.

### The Extract Modulates Mechanical Hyperalgesia and Dynamic Allodynia in Rats

Compared to the sham group, an increase in the scores of mechanical hyperalgesia (withdrawal time of injured hind paw) and dynamic allodynia was observed in CCI group following the surgery (Figures 2A,B). This significant increase in the dynamic allodynia scores was attenuated when rats were administered the two studied dose levels of the extract on days 7 and 14 after the surgery. The low dose level did not show a significant effect on mechanical hyperalgesia on day 7 but exerted a significant reduction in the scores on day 14 following the surgery (Figure 2A). Noteworthy, the extract (400 mg/kg) has a greater effect than pregabalin against mechanical hyperalgesia on day 7, while both dose levels exerted a greater effect than pregabalin on days 7 and 14 against dynamic allodynia.

**FIGURE 2:** Mechanical hyperalgesia and mechanical dynamic allodynia on days 7 and 14 after CCI. Data are expressed as mean ± SEM (n = 6/group). Data were analyzed with RM-ANOVA, and Tukey post hoc test. *, ^#^ and ^@^ denote *p* < 0.05 from sham, CCI and pregabalin, respectively.

### The Extract Attenuates the Structural Derangements of Sciatic Nerve and Brainstem Induced by Sciatic Nerve CCI in Rats

Microscopic examination of H and E-stained transverse sections in the sciatic nerve tissues obtained from the different studied groups is shown in Figure 3 (A-F). Control and sham groups exhibited normal histological appearance, where closely packed nerve fibers of the nerve fascicle were observed. Axoplasm surrounded by unstained area of dissolved myelin was noticed in myelinated nerve fibers. Schwann cells nuclei appeared in-between the nerve fibers and an infrequent endoneurial blood vessel was detected as well (Figure 3A, B). On the other hand, disorganized nerve fascicles with wide separation between most of the nerve fibers were detected in the CCI group along with degenerated nerve fibers (Figure 3C). In pregabalin-treated group, partial restoration of the normal architecture of the nerve vesicle was achieved, as most nerve fibers were intact with only slight separation between them (Figure 3D). Notably, sections from rats treated with the low dose of the extract showed mild improvement in the architecture of the nerve vesicle and nerve fibers (Figure 3E). However, administration of the extract’s high dose resulted in normal nerve fascicle composed of myelinated nerve fibers and Schwann cells nuclei in endoneurial spaces with only slight separation between the nerve fibers (Figure 3F).

**FIGURE 3:** Microscopic representative images of the sciatic nerve transverse sections from the different studied groups **(A)** control group; **(B)** sham group **(C)** CCI group; **(D)** CCI + pregabalin, **(E)** CCI + *P. perfoliatus* extract (200 mg/kg, p.o) **(F)** CCI + *P. perfoliatus* extract (400 mg/kg, p.o). Arrow, bifid arrow, arrowhead, star, and circle illustrate axoplasm, area of dissolved myelin, Schwann cells nuclei, wide separation between the nerve fibers, and degenerated nerve fibers, respectively. (bc) blood vessel, and (bc*) dilated blood vessel. Scale bar, 50 μm x400.

Microscopic examination of H and E-stained brainstem tissues of the different studied groups is shown in Figures 4A–F. Both control and sham groups showed normal neurons, which had vesicular prominent nuclei and basophilic cytoplasm. The acidophilic neuropil contained glial cells with either dark or light stained nuclei (Figures 4A,B). In contrast, most of the neurons from the CCI group were degenerated with shrunken deeply stained nuclei and vacuolated cytoplasm. Some other neurons had irregular deeply stained elongated nuclei with vacuolated cytoplasm. Glial cells were also observed with either lightly or deeply stained nuclei. Moreover, perineural glial cells were seen in close relation to some degenerated neurons (Figure 4C). In the group treated with pregabalin, some neurons were still degenerated with pyknotic nuclei while other neurons were normal (Figure 4D). The group treated with the low dose of the extract (200 mg/kg) revealed still some degenerative changes of the neurons (Figure 4E). However, the use of the higher extract dose (400 mg/kg) partially reversed the degenerative changes, where most neurons were normal, and just few of them showed deeply stained nuclei (Figure 4F). Notably the latter effect was superior to that of pregabalin.

**FIGURE 4:** Microscopic images of brainstem tissues from the different studied groups **(A)** control group **(B)** sham group; **(C)** CCI group **(D)** pregabalin group; **(E)** *P. perfoliatus* extract (200 mg/kg, p.o.) **(F)** *P. perfoliatus* extract (400 mg/kg, p.o.). Arrow, arrowhead, bifid arrow, wavy arrow, and (*) represent normal neurons with flame elongated dark nuclei, neurons with dark stained nuclei and vacuolated cytoplasm, perineural glial cell nuclei, and neuropil respectively. (bc) normal blood capillary, (*bc) dilated blood capillary, (lg) lightly stained glial cell nuclei, (dg) deeply stained glial cell nuclei. Scale bar, 50 μm x400.

### Effect on Apoptosis in Sciatic Nerve

To evaluate the apoptotic status in sciatic nerve, the immunohistochemical staining with anti Bax antibody was carried out to detect the apoptotic cells in all studied groups. As shown in Figure 5, Bax-positive apoptotic cells in sciatic nerve were hardly detected in the control and sham groups (Figures 5A,B). On the contrary, abundant Bax positive apoptotic cells were detected in the CCI groups that received the vehicle (Figures 5C,E). However, the latter response was attenuated in a dose dependent manner with the maximum effect observed in the rats treated with the high dose of the extract (400 mg/kg) that showed 88.5% reduction in the area percent of Bax-positive cells per section. Notably, the effect of the high dose was superior to that of pregabalin, which showed 75.7% reduction in the positive area (Figures 5D,F,G).

**FIGURE 5:** Microscopic images identify the immunoreactivity of the apoptotic marker Bax in the sciatic nerve from the different studied groups **(A)** control group; **(B)** sham group **(C)** CCI group; **(D)** CCI + *P. perfoliatus* extract (Pot, 200 mg/kg, p.o) **(E)** CCI + *P. perfoliatus* extract (Pot, 400 mg/kg, p.o) **(F)** CCI + pregabalin. Scale bar; 50 μm. **(G)** Bar chart showing changes in the area percent of Bax positive cells of the siatic nerve in all different studied groups. The area percent of immuno-positive cells were estimated from six animals/group in perceptive fields at ×400 magnification. One-way ANOVA was used for statistical analysis followed by a post-hoc Tukey test. Values are presented as means ± SEM.*p < 0.05 vs control group; ^#^ *p* < 0.05 vs CCI; ^@^ *p* < 0.05 vs pregabalin.

### Effect on CD68 in Sciatic Nerve

In order to assess the influence of CCI on the macrophages’ infiltration into the sciatic nerve, the expression of the macrophages marker CD68 was evaluated by immunohistochemistry. The control and sham groups displayed few expressions of CD68 positive cells. However, abundant CD68 positive cells were observed in rats exposed to CCI. On the contrary, low dose of the extract exhibited less CD68 positive cells than the CCI group but still revealing a significant difference from the control group. Increasing the dose of the extract to 400 mg/kg abrogated the CCI-mediated increase in the number of CD68 positive cells and demolished, as well, the area percent of CD68 immunoexpression. Notably, this effect was superior to that of pregabalin (Figures 6A–F).

**FIGURE 6:** Microscopic images identify the immunoreactivity of CD68 in the sciatic nerve from the different studied groups **(A)** control group; **(B)** sham group **(C)** CCI group; **(D)** CCI + *P. perfoliatus* extract (Pot, 200 mg/kg, p.o) **(E)** CCI + *P. perfoliatus* extract (Pot, 400 mg/kg, p.o) **(F)** CCI + pregabalin. Scale bar; 50 μm. **(G,H)** Bar charts showing changes in the number of CD68 positive cells and the area percent of CD68 immunoexpression, respectively that were measured from six animals/group in perceptive fields at ×400 magnification. One-way ANOVA was used for statistical analysis followed by a post-hoc Tukey test. Values are presented as means ± SEM.*p < 0.05 vs control group; ^*#*^ *p* < 0.05 vs CCI; ^@^ *p* < 0.05 vs pregabalin.

### Effect on Bcl-2 and Bax in Brainstem

To assess the apoptotic status in the brainstem tissues following CCI induction, the immunohistochemical staining with anti-Bcl-2 and anti-Bax were carried out to detect the antiapoptotic and apoptotic responses, respectively in all the studied groups. Bcl-2-positive cells were mainly detected in the cytoplasm of normal neurons, while Bax-positive cells were detected in the cytoplasm of the degenerated neurons, Figure 7A–F and Figure 8A–F, respectively. Positive Bcl-2 immunoreactivity was obviously observed in the control and sham group (Figures 7A,B) and infrequently demonstrated in the CCI groups that received either no treatment or low dose of the extract (Figures 7C,E). However, CCI groups that received either pregabalin or the higher dose of the extract showed higher Bcl-2 immunoreactivity and most of the neurons showed positive Bcl-2 staining (Figures 7D,F). These results were confirmed by morphometrical and statistical analysis, where the number of Bcl-2-positive cells per section was significantly decreased in the CCI and CCI + low extract dose groups and significantly increased in CCI + pregabalin and CCI + high extract dose groups compared to those in the control and sham groups (Figure 7G). On the other hand, the Bax-positive apoptotic cells were hardly detected in control and sham groups (Figures 8A,B). In contrast, abundant Bax-positive apoptotic cells were detected in the CCI groups (Figure 8C). The latter effect was significantly attenuated in the CCI rats treated with both doses of the extract (400 mg/kg) and was comparable to pregabalin (Figures 8D–F).

**FIGURE 7:** Microscopic images identify the immunoreactivity of the antiapoptotic marker Bcl-2 in brainstem neuronal cells in the different studied groups **(A)** control group; **(B)** sham group **(C)** CCI group; **(D)** CCI + *P. perfoliatus* extract (Pot, 200 mg/kg, p.o) **(E)** CCI + *P. perfoliatus* extract (Pot, 400 mg/kg, p.o) (F) CCI + pregabalin. Arrowhead indicates dark brown staining of the cytoplasm of immuno-positive normal neurons and arrow indicates the negative immunostaining of the affected neurons. Scale bar, 50 μm × 400. **(G)** Bar chart presenting the quantification of the number of Bcl-2-positive normal neurons in all different studied groups. The immuno-positive neurons were counted from six animals/group in perceptive fields at ×400 magnification. One-way ANOVA was used for statistical analysis followed by a post-hoc Tukey test. Values are presented as means ± SEM.*p < 0.05 vs control group; ^#^ *p* < 0.05 vs CCI; ^@^ *p* < 0.05 vs pregabalin.

**FIGURE 8:** Microscopic images identify the immunoreactivity of the apoptotic marker Bax in brainstem neuronal cells in the different studied groups **(A)** control group; **(B)** sham group **(C)** CCI group; **(D)** CCI + *P. perfoliatus* extract (Pot, 200 mg/kg, p.o) **(E)** CCI + *P. perfoliatus* extract (Pot, 400 mg/kg, p.o) **(F)** CCI + pregabalin. Arrow refers to dark brown staining of the cytoplasm of immuno-positive affected brainstem neurons and arrowhead refers to the negative immunostaining of the normal brainstem neurons. Scale bar, 50 μm × 400. **(G)** Bar chart presenting the quantification of the number of Bax-positive normal neurons in all different studied groups. The immuno-positive neurons were counted from six animals/group in perceptive fields at ×400 magnification. One-way ANOVA was used for statistical analysis followed by a post-hoc Tukey test. Values are presented as means ± SEM.*p < 0.05 vs control group; ^#^ *p* < 0.05 vs CCI.

### Molecular Docking Showed That the Components of the Extract Were Able to Bind at the Bcl-2: BH3 Interface

To investigate, on a molecular level, the anti-apoptotic potential of the major phytoconstituents identified in the extract, we docked these compounds at the Bcl-2: BH3 interface. It is well known that the BH3 domain of the pro-apoptotic Bim protein forms a dimer with Bcl-2 by binding at this interface leading to inactivation of Bcl-2. Table 1 shows the docking score (kcal/mol) that relates to the free binding energy of the compounds upon binding to the protein. Apart from caffeic acid glucoside and the carboxylic acids of small molar volume that showed weak binding at Bcl-2: BH3 interface (manifested as high binding energy), the rest of the compounds showed moderate free binding energy ranging from—10.44 to—13.05 kcal/mol (Table 1). This reveals their ability to compete at the Bcl-2: BH3 interface and thus could prevent the dimerization between Bim and Bcl-2. Noteworthy, the iridoid glucoside catalpol sulphate showed the best binding at the interface with minimum free energy of—13.05 kcal/mol.

**TABLE 1:** Docking scores (kcal/mol) of *P. perfoliatus* phytoconstituents at Bcl-2: BH3 interface.

Compound*	Score function (kcal/mol)
	4B4S
Catalpol sulphate	−13.05
*p*-Hydroxybenzoic acid	−7.67
Phloretic acid	−7.92
Catalpol	−10.44
Luteolin 7-glucoside	−10.86
Caffeic acid glucoside	−8.44
Rosmarinic acid	−11.00
Caffeic acid 3-sulfate	−11.10
Phloretic acid sulphate	−10.51

*Previously described from our extract (Rezq et al., 2021). The same extract from Rezq et al. (2021) was used in this study.

### Effect on CD68 and GFAP Expression in Brainstem

In order to evaluate the compensatory mechanism of the glial cells to the brain injury following CCI, the expressions of both microglial marker CD68 and astrocytes marker GFAP were assessed in brainstem sections to detect microgliosis and astrogliosis, respectively. As shown in Figure 9, the control and sham groups exhibited few CD68 positive microglial cells immuno-expression. Abundant CD68 positive microglial cells immuno-expression, on the other hand, was observed in CCI groups that received the vehicle. On the contrary, CCI rats treated with both doses of the extract attenuated CCI-induced microglial activation in a dose dependent manner (Figures 9A–E). The latter effect involved reduction in both the number and area (size) of CD68 positive cells (Figure 9G, H). Notably, the effect of the extract’s high dose was comparable to that of pregabalin (Figures 9E–H). The control and sham groups showed astrocytes that were small with few and short thin processes (Figures 9A,B). On the other side, CCI groups that received the vehicle and low extract’s dose (200 mg/kg) exhibited an increased number of GFAP-immuno-stained astrocytes (4.8- and 2.6-fold, respectively) that were also larger with long thick multiple processes, indicating both astrogliosis and activated glia (Figure 10 C, D, G, H). However, CCI rats treated with the higher extract’s dose (400 mg/kg) or pregabalin showed mild expression of GFAP-immuno-stained astrocytes with short thin multiple processes and overall reduction in both the astrocytes total number (69.2%) and area percent of GFAP immunoreactivity (73.6%, Figures 10E–H).

**FIGURE 9:** Microscopic images identify the immunoreactivity of the microglial marker CD68 in the brainstem of different studied groups **(A)** control group; **(B)** sham group **(C)** CCI group; **(D)** CCI + *P. perfoliatus* extract (Pot, 200 mg/kg, p.o) **(E)** CCI + *P. perfoliatus* extract (Pot, 400 mg/kg, p.o) **(F)** CCI + pregabalin. Arrowheads refer to the dark brown microglial cells. Scale bar; 50 μm. **(G,H)** Bar charts showing changes in the number of CD68 positive cells and the area percent of CD68 immuno-expression, respectively that were measured from six animals/group in perceptive fields at ×400 magnification. One-way ANOVA was used for statistical analysis followed by a post-hoc Tukey test. Values are presented as means ± SEM. *p < 0.05 vs control group; ^#^ *p* < 0.05 vs CCI.

**FIGURE 10:** Microscopic images identify the immunoreactivity of the astrocyte marker GFAP in brainstem in different studied groups **(A)** control group; **(B)** sham group **(C)** CCI group; **(D)** CCI + *P. perfoliatus* extract (Pot, 200 mg/kg, p.o) **(E)** CCI + *P. perfoliatus* extract (Pot, 400 mg/kg, p.o) **(F)** CCI + pregabalin. Arrow refers to the astrocytes with thick branching and over expression of GFAP and arrowhead refers to the thin branching astrocytes. Scale bar; 50 μm. **(G,H)** Bar charts showing changes in the area percent of GFAP-immuno-expression and the number of GFAP-positive cells, respectively (G) Bar chart showing the difference in the area percent of GFAP-immuno-expression in all studied groups that were measured from six animals/group in perceptive fields at ×400 magnification. One-way ANOVA was used for statistical analysis followed by a post-hoc Tukey test. Values are presented as means ± SEM.*p < 0.05 vs control group; #*p* < 0.05 vs CCI.

### The Extract Attenuates Oxidative Stress Caused by Sciatic Nerve CCI in Rats

To investigate the extract’s effect on the CCI induced oxidative stress, the levels of the oxidative stress marker (NOX-1) and the antioxidant enzyme (catalase) were measured in both sciatic nerve and brainstem 14 days following the surgery. It was shown that NOX-1 level was increased in the CCI rats’ sciatic nerves and brainstems (Figure 11A). On the other hand, catalase activity was decreased in both tissues in the CCI group compared to the sham group (Figure 11B). The extract at both dose levels was able to improve the oxidative status in the sciatic nerve and brainstem through decreasing NOX1 levels and increasing catalase activity compared to the CCI group (Figure 11). While the effect of the extract on NOX-1was comparable to that of pregabalin, the latter was more effective to restore catalase activity compared to the extract at its two tested doses (200 and 400 mg/kg).

**FIGURE 11:** Oxidative stress (evaluated with respect to NOX-1, A and catalase, B) in the sciatic nerve and brainstem on day 14 after the surgery. Data (n = 5) are expressed as means ± SEM. Data were analyzed with One-way ANOVA and Tukey test. *, ^#^ and ^@^ denote *p* < 0.05 from sham, CCI, and pregabalin, respectively.

### The Extract Attenuates Neuro-Inflammation Caused by Sciatic Nerve CCI in Rats

To evaluate the effect of the extract on neuro-inflammation, the levels of the pro-inflammatory markers PGE2, TNF-α and NF-κB in addition to the levels of COX-2 and 5-LOX enzymes and the nitrosative stress enzyme iNOS were measured in sciatic nerve and brainstem 14 days following the surgery. Our results showed that all the previously mentioned parameters were elevated in CCI rats relative to the sham group. Both extract’s doses (200 and 400 mg/kg) were able to attenuate the inflammatory response after 14 days of the treatment when compared to the CCI control group. Noteworthy, the extract, especially the high dose, was superior to pregabalin in all the studied pro-inflammatory marker proteins and showed comparable effects to pregabalin on the inflammatory enzymes and iNOS (Figure 12).

**FIGURE 12:** Pro-inflammatory markers and inflammatory enzymes levels in the sciatic nerve and brainstem on day 14 after the surgery. **(A)** PGE2, **(B)** TNF-α, **(C)** NF-κβ, **(D)** iNOS, **(E)** COX-2, and **(F)** 5-LOX in sciatic nerve and brainstem tissues. Data (n = 5) are expressed as means ± SEM. Data were analyzed with One-way ANOVA and Tukey test. *, ^#^ and ^@^ denote *p* < 0.05 from sham, CCI, and pregabalin, respectively.

## Discussion

Chronic neuropathic pain is caused by either neuropathy or illness. It results in abnormal spontaneous exaggerated responses to painful stimuli (hyperalgesia), non-painful stimuli (allodynia), thermal hypersensitivity in addition to the chronic pain sensation (Vasudeva et al., 2014). There are few effective treatments available for managing neuropathic pain. However, currently available medicines have several reported adverse effects and are with subpar efficiency to manage neuropathic pain and only help around half of patients, leaving neuropathic pain therapy a significant unmet medical need. We showed previously that *P. perfoliatus* extract possesses potent analgesic and anti-inflammatory effects. Therefore, the goal of this study was to investigate *P. perfoliatus* extract influence on neuropathic pain and the possible mechanisms behind it.

The major findings from this work on neuropathic pain in rats were 1) *P. perfoliatus* extract attenuated both hyperalgesia and allodynia better than pregabalin on days 7 and 14 days after the surgery 2) treatment with the high extract’s dose reversed the degenerative changes of the sciatic nerve and other degenerated neurons and attenuated as well the glial activation in brainstem with a superior effect to pregabalin 3) the extract mitigated apoptotic changes of both sciatic nerve and brainstem, especially the high dose level 4) the extract suppressed microgliosis and astrogliosis induced by CCI in brainstem 5) the extract attenuated oxidative and nitrosative stress and mitigated neuroinflammation in sciatic nerve and brainstem.

Neuropathic pain was induced in this study by sciatic nerve chronic constriction injury. This model is a reproducible, extensively used, and reliable animal model of chronic neuropathic pain (Dowdall et al., 2005). The CCI injury is associated with injury of the sensory afferents to the foot and with pain hypersensitivity of the hind paw that could last for up to 1 month after the surgery (Austin et al., 2012). Our observations revealed that hyperalgesia and allodynia developed 7 days and became evident 14 days following the surgery. The extract increased the heat withdrawal latency and decreased the scores of mechanical hyperalgesia especially at the high dose level, which showed better effect than pregabalin. It also decreased both cold and dynamic allodynia scores and was superior to pregabalin in these regards. These pain-related behaviors were associated with sciatic nerve structural derangement represented as areas of decreased myelination and nerve fibers degeneration. There are three major types of primary afferent fibers, which are the unmyelinated C, the small diameter, and large diameter myelinated Aβ-fibers. Under normal conditions, pain transmission usually occurs via the nociceptors of C and Aδ fibers, however upon peripheral nerve injury the highly myelinated Aβ fibers are hyper-sensitized and get more involved in sciatic nerve injury-associated allodynia (Basbaum and Fields, 1984). Normally, GABAergic neurons in laminae I-III of the spinal cord and in the ventral brainstem exert inhibitory effect on the Aβ-fibers (Agostinelli and Bassuk, 2021). Synaptic inhibition mediated by both glycinergic and GABAergic receptors at the dorsal horn of the spinal cord and in the related brainstem sites is deteriorated by many mechanisms evoked by peripheral inflammation or nerve injury (Agostinelli and Bassuk, 2021; Xing et al., 2021; Zeilhofer et al., 2021). The loss of GABAergic signaling following neuropathy could explain the hyper-stimulation of the Aβ-fibers that accompanies sciatic nerve injury, a process known as central sensitization (Kocot-Kępska et al., 2021). Moreover, the local nerve injury results in inflammatory hypersensitivity that can lead to phenotype switching of the Aβ fibers to resemble pain fibers. Therefore, synaptic transmission in the spinal cord is enhanced, and the response to innocuous stimuli is exaggerated (Neumann et al., 1996).

To explore further the molecular mechanism beyond the chronic neuropathic pain and the effects of the extract, we assessed the proteins involved in the cascade of events linked to neuropathic pain development. This cascade includes excitotoxicity, oxidative stress, neuro-inflammation and apoptosis (Komirishetty et al., 2016). Following chronic constriction of sciatic nerve and reduction of epineural blood flow, activated Schwann cells, fibroblasts and damaged nerve synthesize and release inflammatory cytokines, chemokines, substance P, prostanoids, and neurotrophic factors (Cui et al., 2000). This is followed by recruitment of immune cells to the site of injury and to the neuronal cell bodies in the dorsal root ganglia, which produce more pro-inflammatory cytokines, chemokines, trophic and growth factors (Saleem et al., 2019). Our results showed that both pro-inflammatory mediators (TNF-α, NF-κB and PGE2) and inflammatory enzymes, COX-2 and 5-LOX were increased in sciatic nerve and brainstem 14 days following the surgery. This indicated more distant effect of sciatic nerve CCI on the brainstem. The extract attenuated, dose dependently, the levels of both pro-inflammatory mediators and inflammatory enzymes in the sciatic nerve and brainstem with a superior effect to pregabalin 14 days following the surgery.

Our interest to study the brainstem is because of its well-established role in neuropathic pain pathology. Multiple studies reported functional alterations in the endogenous pain-modulation system of brainstem to be associated with the chronic progression of neuropathic pain. Additionally, the brainstem is rich in nuclei that are involved in pain transmission including locus coeruleus in the pons, RVM in the medulla, and ventrolateral periaqueductal gray (vlPAG) of the midbrain (Varghese et al., 2014). It is reported that hyperexcitability of CNS neurons or central sensitization resulting from neuro-inflammation following a peripheral nerve injury, is responsible for the development of neuropathic pain and that apoptosis is implicated in central sensitization (DeLeo et al., 2000). One of the most important pro-inflammatory mediators that increased in the injured sciatic nerve and brainstem in our study is TNF-α. It is believed to be released from the recruited inflammatory cells that infiltrate injured sciatic nerve and from microglia in the CNS (Liu et al., 2007). In accordance with our findings, previous studies showed that TNF-α levels also increase in the brain specifically in the locus coeruleus of brainstem and hippocampus of chronic constriction injury (CCI) rats (Ignatowski et al., 1999; Covey et al., 2000). TNF-α binds to two types of TNF-α receptors, type 1 which is responsible for development of apoptosis and type 2 which is linked to the translocation of NF-κB to nucleus and gene expression. The NF-κB is required for the maximal expression of numerous cytokines, including TNF-α and iNOS (Andrade et al., 2011). Thus, TNF-α binding to TNF receptors increases NF-κB which in turn increases its gene expression and promotes for inflammation. Furthermore, it is reported that CCI stimulates local iNOS expression in macrophages and activates Schwann cells within and distal to the injury site. Increased expression of iNOS is associated with increased NO production and nitrosative stress, which contributes to neuropathic pain. The studied extract mitigated the increased iNOS level only in the brainstem with a comparable effect to pregabalin, which also suppressed iNOS in sciatic nerve. Our results indicate that increased iNOS in sciatic nerve is not the key player in neuropathic pain as the extract suppressed hyperalgesia and allodynia and Wallerian degeneration of sciatic nerve without exerting significant effect on sciatic nerve iNOS.

Recruited hematogenous macrophages at the injured sciatic nerve upregulate the expression of COX-2 leading to increasing the production of PGE2 that contributes to the inflammatory response (Ma and Quirion, 2005). After 14 days of the surgery, our results revealed increased COX2 and PGE2 levels in the sciatic nerve and brainstem, which were both suppressed by the extract at the two sites by the end of the experiment. The effect on PGE-2 was dose dependent, and the high dose of the extract was shown to be superior to pregabalin. Previous studies reported that PGE2 was increased in the injured nerves and ipsilateral dorsal root ganglia (DRG) 10 days after CCI. They showed that nerve-injury- and TNF-α-induced pain-associated behavior partly followed the peripheral prostaglandins production (Schäfers et al., 2004).

Besides COX-2 enzyme increased level, we observed increased 5-LOX level in the injured sciatic nerve and brainstem 14 days after the surgery, an effect that was attenuated by the extract. The enzyme 5-LOX is reported to play an essential role in the pathophysiology and the management of neuropathic pain as well. We showed previously that the extract has direct inhibitory effect on COX-2 and 5-LOX *in vitro*. During the development of neuropathic pain, 5-LOX is altered ipsilaterally in both the DRGs and the lumbar spinal cord suggesting that it may influence nociceptive processing (Malek et al., 2014). Suppression of 5-LOX by the extract may play a role in its anti-nociceptive effect. The 12/15 5-LOX and COX-2 enzymes are responsible for the degradation of the endogenous endocannabinoid, anandamide (AEA) producing active AEA metabolites which contribute to the neuropathic pain (Malek et al., 2014). Thus, 5-LOX inhibitors could be potential therapeutics targeted to relief the neuropathic pain-associated symptoms via inhibiting the production of leukotrienes (LTs) which are essential inflammatory mediators in the pathophysiology of neuropathy (Masamichi et al., 2009).

Oxidative stress plays a vital role in the development of neuropathic pain following CCI (Sobeh et al., 2019). Our previous studies showed that antioxidants were able to mitigate the neuropathic pain caused by CCI (Sobeh et al., 2019, 2020; Rezq et al., 2020). Our results showed that the sciatic nerve CCI was associated with an increased level of the oxidative stress enzyme, NOX-1 and decreased antioxidant catalase activity in the sciatic nerve and brainstem 14 days after the surgery. These changes were suppressed by the extract and pregabalin. The antioxidant effects of the extract could be related to its high content of phenolic acids, such as caffeic acid glucoside phloretic acid gallate, syringic acid, caffeic acid sulphate and p-hydroxy benzoic acid (Rezq et al., 2021).

Schwann cells, which may express NOX1, NOX2, and NOX4 mRNAs, were reported to increase only the NOX1 protein levels (De Logu et al., 2017). NOX-1 is important mediator of oxidative stress-induced neuropathic pain via activation of the nociceptor transient receptor potential ankyrin 1 (TRPA1). In addition, NOX-1 activation induces H_2_O_2_ release, which targets TRPA1. It maintains allodynia, by acting on the adjacent nociceptor nerve fibers in a paracrine manner. Silencing or inhibiting NOX1 in Schwann cells reduced nerve injury-induced macrophage infiltration, oxidative stress, and allodynia. It was also reported that NOX1 inhibitors, but not NOX2 or NOX4, reduced neuroinflammation and allodynia (De Logu et al., 2017).

Macrophages quickly travel across the perineurium to penetrate the injured nerve trunk, because of the oxidative stress gradient created by Schwann cells, which in turn release more free radicals. Free radicals damage the peripheral nerves and cause hyperexcitability in the afferent nociceptors, which, in combination with central sensitization, causes spontaneous impulses to be generated inside axons and dorsal root ganglions, contributing to the manifestation of neuropathic pain (Shahid et al., 2021). It is also reported that NOX-1 is expressed in neurons (McCann et al., 2008) and microglia of the CNS (Pendyala and Natarajan, 2010), which is confirmed in our study by its elevation in brainstem of CCI rats. The use of the non-specific NOX inhibitor apocynin or deletion of the p47PHOX subunit inhibited NOX activation in microglia, which did not only decrease the inflammatory responses but also polarized the microglia into the M2 or alternate activation phenotype (Choi et al., 2012).

Previous studies showed that spinal microglial and astrocytes activation and the subsequent increase in the expression of CD68 and GFAP, respectively occurs in the spinal cord 7 days after the CCI surgery (Li et al., 2013; Nishihara et al., 2020). However, microglial and astrocytes activation at the brainstem level is less well elucidated. In this study, we evaluated the responses of two types of glial cells, the microglial cells and the astrocytes in the brainstem 14 days after CCI. Our findings showed that both microglia and astrocytes are activated in brainstem indicated by the increase in CD68 and GFAP expression, respectively. The expression of CD68 and GFAP was suppressed by the high dose of the studied extract. Activated glial cells are involved in the phagocytic destruction of the synapses or the synaptic stripping at higher centers level. Our results are in accordance with a previous study that showed that glial activation and GFAP expression is increased in the thalamus and midbrain after CCI injury (Giardini et al., 2017). Another study revealed that the inhibition of the microglia activity through minocycline administration reduced the hypersensitivity manner of the rats in CCI model (Mika et al., 2009).

Apoptosis and oxidative stress play a role in the onset and progression of neuropathic pain (Areti et al., 2014). Apoptotic changes in the spinal cord following CCI is well documented (Giardini et al., 2017; Liao et al., 2021). In our study, we assessed the apoptotic changes of the sciatic nerve and the neurons of brainstem 14 days after CCI. We observed that the expression of the apoptotic marker, Bax in the sciatic nerve and brainstem was increased 14 days following the surgery. This was associated with a reduction in the antiapoptotic marker, Bcl-2 expression in brainstem. The extract was able to suppress, dose dependently, the Bax expression in sciatic nerve and brainstem. Expression of Bcl-2 in the brainstem was increased by the high dose only. The high dose showed similar effects to pregabalin. This could explain the dose dependent inhibition of allodynia and hyperalgesia of the extract. It was reported previously that the drugs able to inhibit caspase activity and hence apoptosis in the spinal cord have alleviated mechanical allodynia in rats with spared nerve injury (Scholz et al., 2005).

The observed results might be attributed to the presence of several phenolic acids (p-coumaric acid, p-hydroxybenzoic acid, syringic acid and rosmarinic acid), flavonoids (luteolin glucoside, quercetin glucoside) and the iridoid (catalpol sulphate) (Rezq et al., 2021). Comparable neuroprotection activities were observed from polyphenolic rich extracts such as *Thymus fontanesii*, *Thymus algeriensis*, *Haematoxylon campechianum,* and *Salix tetrasperma* (Sobeh et al., 2019, 2020; Rezq et al., 2020).

## Conclusion

Our findings showed that *P. perfoliatus* extract confers neuroprotection against sciatic nerve CCI through multiple signaling pathways, including suppression of apoptosis and glial cells activation, and inhibition of pro-inflammatory cytokines, oxidative and nitrosative stress. The involvement of both peripheral and central mechanisms in *P. perfoliatus*-mediated attenuation of neuropathic pain pathophysiology both on the behavioral and molecular levels highlights it as a multipotent promising agent for the management of neuropathic pain. Further experiments are required to explore the effects of the extract on the dorsal root ganglia and spinal cord as well. Also, future studies are needed to isolate the individual components of the extract and investigate their activities *in vivo* and directly assess the involved mechanisms. In addition, because we employed an experimental CCI animal model for neuropathic pain, we were unable to determine *P. perfoliatus* extract clinical effectiveness (including the appropriate therapeutic dose and treatment time). More research is needed to fully understand the potential and mechanism of action of its analgesic properties. Clinical trials should be done in the future to gain a better understanding of the role of *P. perfoliatus* extract and to investigate whether it has any therapeutic effects in the treatment of neuropathic pain in clinically relevant human individuals.

## Data Availability

The original contributions presented in the study are included in the article/Supplementary Material, further inquiries can be directed to the corresponding authors.
